RETRACTED

# Zizhu Ointment Accelerates Wound-Healing of Diabetic Ulcers through Promoting M2 Macrophage Polarization via Downregulating the Notch4 Signaling Pathway

**DOI:** 10.1155/2022/5173836

**Published:** 2022-05-17

**Authors:** Renyan Huang, Xiaoming Hu, Wenhui Li, Lixiang Wang, Weijing Fan, Qiang Han, Fang Guo, Guobin Liu

**Affiliations:** ^1^Department of Peripheral Vascular Disease, Shuguang Hospital Affiliated to Shanghai University of Traditional Chinese Medicine, Shanghai 201203, China; ^2^School of Life Sciences and Biotechnology, Shanghai Jiao Tong University, Shanghai 200240, China; ^3^Shanghai University of Medicine & Health Sciences, Shanghai 200237, China

## Abstract

**Objective:**

The long-term clinical practice shows that Zizhu ointment (ZZO) is an empirical formula for the treatment of diabetic ulcers (DUs). In this study, we investigated the underlying mechanism of ZZO in the treatment of DU mice.

**Methods:**

Through streptozotocin induction and high-fat diet, a DU mouse model was established and ZZO was given for treatment. The activation of Notch4 signaling was examined by immunofluorescence staining, RT-PCR, as well as Western blotting. Flow cytometry was performed to detect the counts of F4/80+ cells, M1 and M2 macrophages, as well as the expression of CD11c, CD206, etc. The role of Notch4 in wound healing in diabetic mice was verified by Notch4 inhibitors and agonists.

**Results:**

Accelerated wound healing and decreased expression levels of Notch4 and its target genes and ligands were observed in diabetic mice treated with ZZO. ZZO promoted M2 macrophage polarization, downregulated the expression of proinflammatory factors, and upregulated the levels of anti-inflammatory factors. The same tendency was observed in diabetic mice after treatment with Notch4 inhibitors. Knockout of Notch4 accelerated the wound healing rate as well.

**Conclusions:**

ZZO accelerates wound healing of diabetic mice through inhibiting the activation of Notch4 signaling, promoting M2 macrophage polarization, and alleviating inflammation.

## 1. Introduction

Diabetes mellitus (DM) is one of the public health problems, with an estimated 439 million adults (aged 20–79) living with DM worldwide by 2030 [1]. Diabetic ulcer (DU) is one of diabetic complications characterized by delayed wound healing, which decreases the quality of life of diabetic patients and leads to a huge cost. In the United States, the annual cost of treating diabetic wounds is estimated to be $13 billion, which significantly increases the social and economic burden [2–5]. Wound healing is a complex physiological process involving different stages of inflammation, cell proliferation, fibrosis, and remodeling [6]. However, the biological process of diabetic wound healing is interfered and delayed [4, 5], and wounds that remain unhealed for a long time can lead to deterioration and even amputation. Therefore, it is important to develop an effective therapy for treating diabetic wounds with a well characterized molecular mechanism. Zizhu ointment (ZZO) is an empirical formula for the treatment of DUs based on the long-term clinical practice of vascular surgery in our hospital. Its components include Cinnabar (Zhusha), Astragalus mongholicus (Huangqi), Arnebia guttata (Zicao), Donkey hide gelatin (Ejiao), Borneol (Bingpian), and Dragon's Blood (Xuejie). A previous clinical observation of 72 patients with chronic skin ulcer showed that ZZO is effective in the treatment of chronic skin ulcer with a response rate up to 50% [7]. Currently, ZZO is applying for China's invention patent (ZL201010186284.X) as “An external use of Chinese medicine ointment preparation for treating diabetic foot.” ZZO has been proved to be a good treatment for DUs. However, the underlying mechanisms of ZZO in the treatment of DUs have not been clearly elucidated and warrant further exploration. Notch signaling is a conserved signaling pathway that determines cellular differentiation and proliferation as well as survival [8, 9]. The Notch pathway consists of Notch receptors, Notch ligands, and intracellular proteins that act synergistically to transmit signals to the nucleus. The Notch receptors include an intracellular domain, a transmembrane, and an extracellular domain. The Notch ligands include Jagged (Jag1, Jag2) and Delta-like (Dll1, Dll3, Dll4) proteins that can bind to the Notch extracellular domain and induce the intracellular domain release, thus entering the nucleus and activating downstream proteins such as Hes and YRPW motif protein family genes associated with Hes [10]. It is well documented that the Notch signal is involved in the production of cytokines and the regulation of immune responses [11–13]. Xu, H et al. found that Notch-RBP-J, the major nuclear transducer of Notch signaling, enhanced TLR4-induced expression of key mediators of classically activated M1 macrophages [12]. Palaga, T et al. [13] found that Notch signaling is activated by TLR stimulation and regulates the function of macrophages. Therefore, Notch signaling can regulate macrophage-mediated inflammation. Given the crucial role of Notch4 in inflammatory processes, we hypothesized that Notch4 may play an important role in diabetes-related wounding. We also speculated that the mechanism of action of ZZO could be driven through its regulatory effects on Notch4 signaling.

RETRACTED

Therefore, in this study, a mouse DU model was established under the inducement of streptozotocin (STZ) combined with high-fat diet and ZZO was used for treatment, aiming to investigate the role of ZZO in the treatment of diabetic wounds and examine whether the mechanism of action is through the regulation of Notch4 signaling.

## 2. Materials and Methods

### 2.1. Composition and Preparation of ZZO

The main ingredients of ZZO, including Cinnabar, Comfrey, Dragon's Blood, Astragalus, Donkey-hide gelatin, and Borneol pieces, were purchased from Shanghai Kangqiao Chinese Medicine Tablet Co., Ltd, and all met the quality control standards. According to the configuration process, they were processed and produced by Wuhan Ma Yinglong workshop. The ratio of the main ingredients of ZZO to the base materials was 1 : 8, and the ratio of the main medicines (by weight) of Cinnabar, Comfrey, Dragon's Blood, Astragalus, Astragalus, and Borneol was 7 : 3:3 : 6:5 : 1. The excipients of ZZO included poloxamer, propylene, water, glycerol (glycerin), polyethylene glycol (PEG), polyethylene glycol (PEG) 1500, polyethylene glycol (PEG) 4000, and ethyl p-hydroxybenzoate, and the ratio was 34 : 24 : 70 : 2.6 : 9:9 : 3:0.06.

### 2.2. Establishment of a DU Mouse Model

All wild-type C57BL/6 and Notch4 knocked out mice were purchased from Shanghai Nan fang model Biotechnology Co., Ltd (Shanghai Model Organisms Center, Inc.). The animals were kept in a pathogen-free environment under a 12 : 12-h light-dark cycle, with the humidity and temperature controlled at 60 ± 3% and 25 ± 2°C, respectively, and free access to water and food. To construct a type 2 diabetic mice model, mice were fed with a high-fat diet comprised of 60% calories (D12492, Research Diets, Inc.) for 3 weeks and subsequently injected with an intraperitoneal dose of STZ (40 mg/kg/day) daily for one week. When the level of fasting blood glucose was greater than 250 mg/dl, it was confirmed to be type 2 diabetes. All of the animal experiments were approved by the Animal Ethics Committee of Shanghai University of Traditional Chinese Medicine (Approval No. PZSHUTCM190308012) and were conducted in compliance with Guidelines for the Care and Use of Laboratory Animals.

### 2.3. Construction and Treatment of Excisional Wound Splinting Rat Model

Mice with skin wounds were distributed into five groups of 20 individual mice: (1) control group (*n* = 20) whose nondiabetic mice were administered with phosphate-buffered saline (PBS). (2) Diabetic ulcer group (*n* = 20) whose mice were administered with PBS. (3) Diabetic+ZZ0 group (*n* = 20) which were treated with ZZO at the wound site. (4) Diabetic+inhibitor (DAPT (GSI-IX), 10 mg/kg, 3 weeks, 5 days per week, intraperitoneally) group (*n* = 20). (5) Diabetic+agonist (jagged1, 10 ug/kg, once per week, 3 weeks, intraperitoneally) group (*n* = 20).

RETRACTED

### 2.4. Wound Closure Analysis

The wound healing condition of mice was monitored at day 0, 3, 7, and 14 by capturing the wound area with a camera. The healed wound area was quantified using Image J software (Bethesda, MD) and presented as the percentage calculated by the following formula: 1 – (wound area day *t*_1_/wound area day *t*_0_)]  ×  100%, wherein *t*_0_ = initial time point, and *t*_1_ was the time when the wound healing was assessed.

### 2.5. Haematoxylin-Eosin (HE) Staining

To observe the effect of the ZZO on the liver and kidney, the liver and kidney tissues collected from mice were embedded in paraffin from different mouse models and cut into 4 *μ*m slices. The hematoxylin-eosin (HE) staining was performed after dewaxing of liver sections.

### 2.6. Immunofluorescence (IF) Staining

For IF staining, wound skin tissues collected from the mice were blocked with 5% (m/v) BSA, permeabilized with 0.5% triton X-100, and fixed with 4% paraformaldehyde. Then, the specimens were incubated with Notch4 (1 : 1000) at 4°C overnight, followed by 1 hour of incubation with the Alexa Fluor 488 conjugated secondary antibody at room temperature. The nuclei were then dyed with 4′,6-diamidino-2-phenylindole (DAPI) for 15 minutes. The images were obtained with the use of a confocal microscope (LeicaSP8, Germany).

### 2.7. Isolation and Flow Cytometry of Mice Peritoneal Macrophages

Two milliliters of 3% dehydrated thioglycolic acid medium were injected into mouse abdominal cavity once daily for three days. The mice were killed by the dislocation of the cervical spine, and the skin was cut aseptically to completely expose the peritoneum. Then, 8 ml of serum-free medium was injected to rinse the abdominal cavity of the mouse; this step was repeated three times to collect the abdominal fluid into a 50 ml centrifuge tube. After 5 minutes of centrifugation (1000 rpm), the cell suspension was resuspended in RPMI 1640 containing 10% FBS. Tris NH4Cl was used to lyse the red blood cells. Antibodies against F4/80 BM8 (ab6640, Abcam), CD11c (ab219799, Abcam), and CD206 (PA5-46994, ThermoFisher Scientific, San Jose, CA, USA) were used for the characterization of M1 (F4/80 + CD11c + CD206-) or M2 (F4/80 + CD11c-CD206+) macrophages. Flow cytometry was performed with the use of a FACS Aria flow cytometer.

### 2.8. RNA Extraction and RT-PCR

Total RNA was extracted from frozen skin specimens with RNAiso Plus reagent (Takara, Shiga, Japan) and quantified using NanoDrop 2000 (Thermo Scientific, USA). A 1000 ng aliquot of total RNA was then reverse transcripted to complementary DNA (cDNA) with PrimeScriptTM RT Master Mix (Takara). The kit and instrument used for amplification were FastStart Essential DNA Green Master and LightCycler® 96 instrument (Roche, Basel, Switzerland), respectively. Reaction condition is as follows: 95°C for 10 min, and then 45 cycles of 95°C for 10s, and finally 60°C for 30 s. Actin was used as a reference gene. The relative expression of genes was obtained using the 2^−ΔΔCt^ method.

RETRACTED

### 2.9. Western Blot Assay

Skin tissue samples, stored at −80°C, were homogenized in RIPA lysis buffer with Tissue Lyser II (QIAGEN, Hilden, Germany). Then, after centrifugation at 12000 rpm for 15 min, the BCA protein assay kit was used for protein quantification. Subsequently, proteins were purified on the 10% SDS-PAGE gel (Yamei, China) before transferring to a PVDF membrane for 2 h at room temperature. After blocking in skimmed milk (5%) for 2 h, the membrane was incubated overnight with primary antibodies (1 : 1000) against Notch4, Hes1, and beta-actin at 4°C. The primary antibodies were purchased from Cell Signaling Technology (Danvers, MA, USA). After 3 successive washes (10 min/each time) in TBST, the membrane was incubated with a HRP-conjugated secondary antibody containing antirabbit immunoglobulins G (IgG, 1 : 5000) or mouse anti-IgGs (1 : 5000) at room temperature for 2 h. The ECL kit (GE Healthcare, Milwaukee, WI, USA) was used for signal visualization.

### 2.10. Statistical Analysis

The obtained results were described as the mean ± standard deviation (SD), and graph pad prism (*v*7.0; Graph Pad software Inc. San Diego, California, USA) was used for statistical analysis. The one-way analysis of variance (ANOVA) was used for the detection of significance between groups with a cut-off value of *p* < 0.05.

## 3. Results

### 3.1. ZZO Promotes Wound Healing in Diabetic Mice Induced by STZ

To investigate the effect of ZZO on diabetic wound healing, the wound closure of mice was observed on days 0, 3, 7, and 14. As shown in Figure 1(a), compared with the control group, the wound closure decreased in diabetic mice, while ZZO treatment accelerated wound contraction in diabetic mice. Quantitative results of wound closure rate (the percentage of wound reduced from the initial wound) are shown in Figure 1(a). It was found that the wound closure rate was decreased in diabetic mice, but this was annihilated by the treatment of ZZO (Figure 1(b)). Additionally, HE staining of the liver and kidney (Figure 1(c)) showed no significant changes in both tissues in different groups, which indicated that ZZO treatment had no side effects. These results demonstrated that the treatment of ZZO accelerated wound healing in diabetic mice.

RETRACTED

### 3.2. ZZO Inhibiting the Activation of Notch4 in Skin Tissue of Diabetic Mice

To explore the role of Notch4 in wound healing in diabetes and its potential effect of ZZO treatment on diabetic wounds, we detected the expression level of Notch4 intracellular domain by IF staining, RT-PCR, and Western blotting. As indicated in Figure 2(a), the expression level of Notch4 was activated in the skin of mice with diabetes; this result was further confirmed by the upregulation of Notch target genes (Hey1, Hes1) (Figures 2(b) and 2(c)). Moreover, upregulated Notch ligands Dll4 and Jagged1 were observed in the skin of mice with diabetes (Figure 2(c)); however, the expression level of Notch4 and its target genes and ligands were significantly decreased in the ZZO treatment group, which demonstrated that ZZO can inhibit the activation of Notch4 signaling induced by DUs.

### 3.3. ZZO Treatment Promotes M2 Macrophage Polarization

Furthermore, we investigated whether ZZO could alleviate inflammation in DUs via modulating macrophages. The macrophages were extracted from the mice peritoneum, and F4/80, CD11c, and CD206 antibodies were detected to distinguish the M1 and M2 macrophages; then, we detected the changes of macrophages in each group by flow cytometry. As shown in Figures 3(a) and 3(b), the macrophage count and M1/M2 ratio were increased in the diabetic ulcer group, which was suppressed by ZZO treatment. These results demonstrated that ZZO might promote anti-inflammatory M2 polarization. Furthermore, we detected the levels of proinflammatory (iNOS, TNF-*α*, IL-6, and MCP-1) as well as anti-inflammatory factors (IL-4, IL-10, CD206 and ARG1) by RT-PCR in different groups; as shown in Figures 3(c) and 3(d), ZZO intervention statistically reduced iNOS, TNF-*α*, IL-6, and MCP-1 contents induced by wound in diabetic mice, but increased IL-4, IL-10, CD206, and ARG1 to reduce the inflammation of DUs. This is consistent with the above findings that ZZO accelerates the wound healing of DU mice through promoting M2 macrophage polarization.

### 3.4. Inhibition of Notch4 is Beneficial to the Healing of DUs

To investigate the role of Notch4 protein in the healing of DU mice, we detected the effects of Notch4 inhibitors and Notch4 agonists (Jagged1, JAG1) in DU mice. As shown in Figure 4(a), Notch4 inhibitor (N-[N-(3,5-difluorophenacetyl)-1-alanyl]eS-phenylglycinet-butylester, DAPT) treatment also partly accelerated the wound healing in DU mice, but its effect was inferior to that of ZZO treatment, while no obvious improvement was observed after Notch4 agonist treatment. The quantitative results of wound closure rate on days 0, 3, 7, and 14 in different groups is shown in Figure 4(b), which demonstrated that the inhibition of Notch4 promoted the healing of DUs. Subsequently, we observed the changes of the level of macrophages and the ratio M1/M2 after DAPT and JAG1 treatment. As shown in Figure 4(c), DAPT and JAG1 had no significant influence on the count of macrophages. Next, we detected the levels of proinflammatory (iNOS, TNF-*α*, IL-6, and MCP-1) and anti-inflammatory factors (IL-4, IL-10, CD206, and ARG1) through RT-PCR assay. As shown in Figures 4(d) and 4(e), the Notch4 inhibitor also inhibited TNF-*α*, IL-6, and upregulated IL-10, which demonstrated that the inhibition of Notch4 could partly reduce inflammation in diabetic mice. All these showed that ZZO facilitated wound healing through suppressing the expression of Notch4, which was similar to the effect of the Notch4 inhibitor.

RETRACTED

### 3.5. ZZO Increases Wound Healing of DUs in Mice by Suppressing the Expression of Notch4 and Promoting M2 Macrophage Polarization

To determine whether ZZO promotes wound healing in DU mice by inhibiting Notch4-mediated M2 polarization, we observed the effect of ZZO on mice with Notch4 gene knockout. The level of Notch4 was detected by Western blotting. As shown in Figure 5(a), Notch4 was significantly decreased in the Notch4 knock-out mice. We also observed wound healing in each group and found that the knockout of Notch4 accelerated wound healing, but the effect was not as good as that of the ZZO group. Besides, ZZO had no significant effect on wound healing in Notch4-/-DU mice (Figures 5(b) and 5(c)), which demonstrated that the inhibition of Notch4 was beneficial to wound recovery, and it was not the only mechanism of action for ZZO to accelerate wound healing. For further verification, we determined the changes of macrophage count and M1/M2 ratio in each group. The results showed that the count of F4/80+ cells and the ratio of M1/M2 were significantly increased after the treatment of ZZO (Figures 5(d) and 5(e)). However, in the Notch4 knockout group, these changes were neither found nor affected by ZZO. The levels of proinflammatory (iNOS, TNF-*α*, IL-6, and MCP-1) and anti-inflammatory factors (IL-4, IL-10, CD206, and ARG1) were also detected (Figures 5(f) and 5(g)). ZZO downregulated iNOS, TNF-*α*, IL-6, and MCP-1 and elevated IL-4, IL-10, CD206, and ARG1 in DU mice, but there was no significant difference after ZZO treatment in Notch4 knock-out group. These results indicated that Notch4 was a key protein regulated by ZZO in DUs, and Notch4 knockout counteracted the effects of ZZO on diabetic wounds. These findings indicated that ZZO accelerated the wound healing of DU mice by suppressing the expression of Notch4 and promoting M2 macrophage polarization to alleviate inflammation.

RETRACTED

## 4. Discussion

Diabetic ulcer, as a complication of diabetes mellitus, causes high mortality and disability in diabetic patients. Nonetheless, effective therapy options for this condition are limited. In the present study, ZZO treatment significantly accelerated the wound closure in diabetic mice induced by STZ combined with high-fat diet and reduced inflammation, which may benefit wound healing. In addition, ZZO induced M2 macrophage polarization. Furthermore, we found that the effect of ZZO was mediated by NOTCH4 signaling. The present study is the first to demonstrate that ZZO promotes wound healing in diabetic mice by regulating M2 macrophage depolarization via the NOTCH4 signaling.

ZZO is widely used in traditional Chinese medicine and is known for its therapeutic properties for various diseases. However, scientific studies on this preparation in the treatment of diseases remain limited. So far, no scientific research has yet demonstrated the therapeutic effect of ZZO in diabetes, especially the healing of DUs. This study, for the first time, shows that ZZO is effective in the treatment of DUs. Inflammation, one of the pathological processes associated with DUs [14–17], was effectively inhibited by ZZO as demonstrated by its influences on the expression of multiple markers such as iNOS, TNF-*α*, IL-6, MCP-1, IL-4, IL-10, ARG1, and CD206. Macrophage polarization is correlated with inflammation [18–22]. It is shown that promoting M2 macrophage polarization partly inhibits obesity-induced chronic inflammation [23] and diabetic wound-healing [24–27]. Therefore, we detected the levels of M1 and M2 macrophage polarization with specific markers. The results identified enhanced M2 macrophage polarization, upregulated anti-inflammatory factors, and reduced proinflammatory factors by ZZO.

Notch pathway participates in the process of DUs and is activated by high glucose levels through the interaction between Notch receptors (Notch 1–4) and ligands; the inhibition of Notch signaling enhanced diabetic wound healing [28]. Here, we report that the Notch pathway was activated in DU mice and that ZZO treatment decreased the expression levels of Notch4 protein, its downstream target genes (Hes1, Hey1), and ligands (Dll4, Jagged1). The Notch4 inhibitor DAPT exerted effects similar to those of ZZO. We also observed the effect of ZZO in mice with Notch4 knockout and found that the wound closure was accelerated but the effect was not as good as ZZO treatment.

Notch pathway is involved in macrophage polarization [12]. To further elucidate the mechanisms of ZZO alleviating DUs, and understand the regulatory function of Notch4 protein in M2 macrophages polarization, Notch4 gene was knocked out in mice to measure macrophage count and M1/M2 ratio. ZZO treatment increased the level of above variables; however, in the Notch4 knockout group, no such change was observed and the effect of ZZO was eliminated. Our research experimentally demonstrates the efficacy of ZZO in diabetic wound healing, deepens our understanding of diabetic wound healing, and supports the development of Notch-based therapies for DUs.

RETRACTED

## 5. Conclusion

In conclusion, ZZO can accelerate wound healing of DUs in mice, which may be attributed to the suppression of the activation of Notch4 signaling pathway, promotion of M2 macrophage polarization, and the inhibition of inflammation. Further elucidation of the underlying mechanism of ZZO on wound healing may provide more convincing evidence for this drug as a therapeutic for DUs.

## Figures and Tables

**Figure 1:** Zizhu ointment promotes diabetic wound healing in STZ-induced diabetes in mice. (a) Representative photos of mice wounds on days 0, 3, 7, and 14 in different groups. (b) The rate of wound closure on days 3, 7, and 14 in different groups. (c) Pictures HE staining of the liver and kidney in different groups. ^*∗∗*^*p* < 0.01 vs control group; ^#^*p* < 0.05 vs diabetic ulcer group; ^##^*p* < 0.01 vs diabetic ulcer group.

**Figure 2:** Zizhu ointment inhibiting the activation of Notch4 in skin tissue of diabetic mice. (a) Immunofluorescence of Notch4 protein in different groups. (b) Western blotting results of Notch1 and Hes1. (c) Quantitative PCR results of Notch4, Hes1, Hey1, dll4, and Jagged1. ^*∗∗*^*p* < 0.01 vs control group; ^#^*p* < 0.05 vs diabetic ulcer group; ^##^*p* < 0.01 vs diabetic ulcer group.

**Figure 3:** Zizhu ointment treatment promotes M2 macrophage polarization. (a) The count of F4/80^+^ cells in different groups. (b) The M1/M2 ratio in different groups. (c) Relative expression of proinflammatory markers IL-6, MCP-1, iNOS, and TNF-*α*. (d) Relative expression levels of anti-inflammatory factors IL-4, CD206, ARG1, and IL-10. Data were expressed as mean ± standard deviation (SD); ^*∗*^*p* < 0.01 vs control group; ^#^*p* < 0.05 vs diabetic ulcer group; ^##^*p* < 0.01 vs diabetic ulcer group.

**Figure 4:** Inhibition of Notch4 is beneficial to the healing of diabetic ulcer. (a) Representative images of wound healing in different treatment groups. (b) Wound closure analyzed on days 3, 7, and 14 by Image J (*n* = 10). (c) The count of F4/80^+^ cells in different groups. (d) The ratio of M1/M2 in different groups. (e) Relative expression of IL-6 MCP-1, iNOS, and TNF-*α*. (f) Relative expression of anti-inflammatory factors IL-4, CD206, ARG1, and IL-10. ^*∗*^*p* < 0.05 vs control group; ^*∗∗*^*p* < 0.01 vs control group; ^#^*p* < 0.05 vs diabetic ulcer group; ^##^*p* < 0.01 vs diabetic ulcer group.

RETRACTED

**Figure 5:** Zizhu ointment accelerates wound healing in diabetic ulcer mice by suppressing the expression of Notch4 and promoting M2 macrophage polarization. (a) Western blotting results of Notch4 in control and Notch4 knockout groups. (b) Representative images of wounds healing after different treatments. (c) Wound closure on days 3, 7, and 14 by Image J (*n* = 10). (d) The count of F4/80^+^ cells in different groups. (e) The ratio of M1/M2 in different groups. (f) Relative expression of IL-6 MCP-1, iNOS, and TNF-*α*. (g) Relative expression of IL-4, CD206, ARG1, and IL-10. ^*∗*^*p* < 0.05 vs control group; ^*∗∗*^*p* < 0.01 vs control group; ^#^*p* < 0.05 vs diabetic ulcer group; ^##^*p* < 0.01 vs diabetic ulcer group.

## Data Availability

The labeled dataset used to support the findings of this study are available from the corresponding author upon request.

## 6. Abbreviations

DM: Diabetes mellitus
ZZO: Zizhu ointment
DU: Iabetic ulcer.
